# Spin Orbit Coupling Gap and Indirect Gap in Strain-Tuned Topological Insulator-Antimonene

**DOI:** 10.1186/s11671-016-1666-4

**Published:** 2016-10-18

**Authors:** Chi-Ho Cheung, Huei-Ru Fuh, Ming-Chien Hsu, Yeu-Chung Lin, Ching-Ray Chang

**Affiliations:** 1 Graduate Institute of Applied Physics, National Taiwan University, Taipei, 10617 Taiwan; 2 Department of Physics, National Taiwan University, Taipei, 10617 Taiwan

**Keywords:** Topological insulator, Large-bulk band gap

## Abstract

Recently, searching large-bulk band gap topological insulator (TI) is under intensive study. Through *k*·*P* theory and first-principles calculations analysis on antimonene, we find that *α*-phase antimonene can be tuned to a 2D TI under an in-plane anisotropic strain and the magnitude of direct bulk band gap (SOC gap) depends on the strength of spin-orbit coupling (SOC) which is strain-dependent. As the band inversion of this TI accompanies with an indirect band gap, the TI bulk band gap is the indirect band gap, not the SOC gap. SOC gap can be enhanced by increasing strain, whereas the indirect band gap can be closed by increasing strain, such that large bulk band gap are forbidden. With the *k*·*P* theory analysis on antimonene, we know how to avoid such an indirect band gap. In case of indirect band gap avoided, the SOC gap could become the bulk band gap of a TI which can be enhanced by strain. Thus our theoretical analysis can help searching large bulk band gap TI.

## Background

In the past 10 years, topological insulator phase has emerged in condensed matter physics with theoretical predictions and experimental observations of this phase in real materials [1–32]. When a material turns into TI phase, it is insulating in the bulk band and conducting on the surface (or edge in two dimensions). The surface states are protected by time reversal symmetry (TRS) and have spin momentum locking property.

Nowadays, the size of manufactured semiconductors almost reaches atomic scale, so it is important to have a breakthrough development in new device operation mechanisms. A utilization of the spin property of electrons is one of the promising venues. Since TI has TRS protected surface states with spin momentum locking property, it could be applied to spintronic devices.

Due to the soaring prices of rare earth materials, narrow bulk band gaps, and stringent ambient condition requirements, TI materials so far available are not practical for industrial production. Thus, searching new TI material or transforming a normal insulator into a topological one are still issues of immediate interest.

Band inversion is a necessary condition for inducing TI phase. Applying strain is one of the methods to cause a band inversion. If spin-orbit coupling (SOC) is ignored, system usually becomes metallic due to the band crossing caused by the band inversion between the highest valence band (VBM) and the lowest conduction band (CBM). SOC is the key to opening a gap (SOC gap) at such crossing point to keep the systems remaining insulating in bulk and meet another necessary condition of inducing TI phase. Furthermore, if TI phase is induced, and the bulk band gap is large enough, such a TI phase continues to exist at room temperature and has a small finite size effect [33] and may become one of the promising candidates of spintronic devices.

The first-principles calculation results of strained *α*-phase antimonene shows that strain not only can induce TI phase on antimonene but also can enhance the magnitude of TI’s direct bulk band gap (SOC gap), such that the magnitude of the SOC gap no longer depends on the atomic order only. We know the reason of this phenomenon is because the strain can enhance the SOC between VBM and CBM, such that the SOC opens a larger band gap in antimonene. Unfortunately, the band inversion accompany with an indirect band gap; thus, the SOC gap is not the bulk band gap of antimonene. Through *k*·*P* theory, we learn that, in an anisotropic system, the band inversion of a TI phase transition will accompany with an indirect band gap if VBM and CBM cannot couple to each other by non-SOC *k*·*P* term.

Such a theoretical and numerical analysis makes it clear how the strain tunes the SOC gap of a TI and the cause of the indirect band gap. It can help applying such a mechanism on other materials to achieve the goal of searching large bulk band gap TI among light atoms to meet the requirement of spintronic devices with low prices.

## Crystal Structure

Our system is a monolayer puckered honeycomb antimonene, which belongs to space group no. 53-Pmna [34–36], and its crystal structure is shown at Fig. 1.

**Fig. 1:** The crystal structure of monolayer antimonene. **a**, **c** The top views of the monolayer. **b** Side profile view. **d** The first Brillouin zone of the monolayer antimonene. The isotropic or anisotropic strain in this paper change lattice constant and the structure parameters, but the crystal structure symmetry remains intact

We have simulated the situations in which antimonene finds itself under an in-plane isotropic compress strain and an in-plane anisotropic strain. The applied strain is defined as $\frac {a-a_{0}}{a_{0}} \times 100~\%$, where *a* and *a*_0_ are the lattice constants for the strained and relaxed structures, respectively. During the relaxation, we force the *x* and *y* direction lattice constants of the unit cell to remain intact, and every atom is free to move to its equilibrium position. Isotropic or anisotropic strain changes lattice constant and the structure parameters, but the crystal structure symmetry remains the same.

## Methods

The first-principles calculations are performed by the Vienna Ab initio Simulation Package (VASP) [37, 38]. We use the generalized gradient approximation (GGA) and the Perdew-Burke-Ernzerhof (PBE) exchange-correlation functional along with the projector-augmented wave potentials for self-consistent total energy calculations and geometry optimization. The critical strain for topological phase transition depends on the band gap of antimonene. In order to avoid underestimating the critical strain, hybrid Heyd-Scuseria-Ernzerhof (HSE)06 method [39] should be used, but as this paper is to give qualitative analysis on SOC gap and indirect band gap of TI instead of quantitative prediction for the critical strain of topological phase transition, therefore (HSE)06 method is not used in our first-principles calculations. The energy convergence criteria for electronic and ionic iterations are set to be 10^−8^ eV. The reciprocal space is meshed at 12 × 16 × 1 using the Gamma-centered grid method. The kinetic energy cutoff for the plane wave basis is 500 eV. In order to simulate a monolayer of antimonene, a unit cell with periodic boundary conditions is used. A vacuum space of 1.2 nm was applied to minimize the interaction between the monolayers.

## Results and Discussion

### Strained Antimonene Without Considering SOC

In this subsection, we analyze the band curvature of strained antimonene with *k*·*P* theory. It is well known that from Schrödinger equation and Bloch wave function, the Hamiltonian for a 2D system can be written in the following form:

1 $$  H_{0}=\frac{\hbar^{2}}{2m_{0}}\left({k^{2}_{x}}+{k^{2}_{y}}\right),  $$

2 $$  H_{k\cdot P}=\frac{\hbar^{2}}{m_{0}}(k_{x}P_{x}+k_{y}P_{y}),  $$

3 $$ H_{SO}=\frac{\hbar}{4{m^{2}_{0}}c^{2}}\bigtriangledown V \times \stackrel{\to }{P} \cdot \stackrel{\to }{\sigma},  $$

4 $$  H_{SO,k}=\frac{\hbar}{4{m^{2}_{0}}c^{2}}\bigtriangledown V \times \stackrel{\to }{k} \cdot \stackrel{\to }{\sigma},  $$

where *k* is the wavenumber, $\hbar $ is the reduced Planck constant, *m*_0_ is the electron rest mass, *c* is the speed of light, *V* is the potential, *P*→ is a momentum operator, *σ* is Pauli matrix, *H*_0_ is the free electron energy dispersion, *H*_*k*·*P*_ is the non-SOC *k*·*P* perturbative terms, *H*_*SO*_ is the *k*-independent SOC perturbative terms and *H*_SO,*k*_ is the k-dependent SOC perturbative terms. Since we have not yet considered the SOC, so *H*_SO_ and *H*_SO,*k*_ are ignored in this subsection.

Here, we present a three-band model, in which the first two bands are the second highest and the highest valence bands, and the third one is the lowest conduction band (under zero strain). The band indices of these three bands are 1, 2, and 3, from the lowest to the highest, respectively. Below is the effective Hamiltonian of the three-band model,

5 $$\begin{array}{*{20}l}  H_{t}&= \left(\begin{array}{lll} <u_{1}|H_{t}|u_{1}>& <u_{1}|H_{t}|u_{2}>& <u_{1}|H_{t}|u_{3}>\\ <u_{2}|H_{t}|u_{1}>& <u_{2}|H_{t}|u_{2}>& <u_{2}|H_{t}|u_{3}>\\ <u_{3}|H_{t}|u_{1}>& <u_{3}|H_{t}|u_{2}>& <u_{3}|H_{t}|u_{3}>\\ \end{array}\right)\\ &= \left(\begin{array}{ccc} A_{11}k^{2}+C_{1} & 0 & 0 \\ 0 & A_{22}k^{2}+C_{2} & A_{23}k_{x} \\ 0 & {A}_{23}^{*}k_{x} & A_{33}k^{2}+C_{3} \\ \end{array}\right), \end{array} $$

where *H*_*t*_=*H*_0_+*H*_*k*·*P*_,*u*_*n*_ is the *Γ* point state wave function of the *n*th band, *A*_*nm*_ is the coefficient of matrix element <*u*_*n*_|*H*_*t*_|*u*_*m*_>, n, m = 1, 2, 3, and *C*_1_,*C*_2_,*C*_3_ are the *Γ* point energy of band 1, 2, 3, respectively.

In Eq. 5, we apply group theory to examine whether or not the matrix element <*u*_*n*_|*O*|*u*_*m*_> of the operator *O* vanishes. This matrix element can be nonzero only if the irreducible representation (IRR) associated with the operator *O* is included in the direct sum decomposition of the direct product of the two IRRs of the basis functions [40–42]. Consequently, band 1 does not couple to band 2 or band 3, but band 2 and band 3 are coupled in *x* direction.

It should be noted that either isotropic or anisotropic strain, which mentioned in “Crystal Structure” section, does not change the symmetry of antimonene, so the form of the effective Hamiltonian does not change either [43]. Thus, we can use the symmetry discussion of space group No.53- *P* *m* *n* *a* to simplify the effective Hamiltonian.

Applying the Löwdin partition to the first order approximation, the energy dispersion relation for each band is

6 $$  E_{nk} \approx H_{nn} + \displaystyle\sum_{\alpha \neq n}\frac{H_{n \alpha}H_{\alpha n}}{E-H_{\alpha\alpha}},  $$

where *E*_*nk*_ is the energy of band *n* with a wavenumber *k*,*E*−*H*_*αα*_ is the energy difference between band *n* and band *α* at *Γ* point. Finally, *H*_*nn*_,*H*_*nα*_, and *H*_*αn*_ are the matrix elements in Eq. 5 with *n*,*α*=1,2,3.

Equation 6 implies that if strain induces band inversion between VBM and CBM, then the second term of the dispersion relation of VBM and CBM changes sign as the energy gap between these two bands changes sign. Consequently, if only *k*_*x*_ term or only *k*_*y*_ term exists in the coupling term of the *k*·*P* Hamiltonian of these two bands, the band curvature of these two bands in one of the directions changes sign after the band inversion while the curvature in another direction remains the same and the band structure of these two bands become saddle shaped, such that there will be a band crossing point between VBM and CBM in one of the *k* directions, as shown in Fig. 2 a. If the coupling term of the *k*·*P* Hamiltonian of these two bands is zero, the curvature of these two bands remains the same, thus there will be a band crossing point between VBM and CBM in each *k* direction, as shown in Fig. 2b.

**Fig. 2:** **a** Band structures with −6,−8,and−10 *%* in-plane isotropic strain. **b** Band structures with different values of in-plane anisotropic strain. *Positive strain* indicates expansion and *negative strain* indicates compression. All energies are referenced to Fermi level. The *dashed lines* are merely a guide for viewing the energy shifts of each band. As band 2 and band 3 are coupled at *k*_*x*_ direction while decoupled at *k*_*y*_ direction, band structure of these two bands become saddle-shaped after band inversion in a way that there is a band crossing point between VBM and CBM in *k*_*y*_ direction. Band 1 and band 3 are decoupled; band inversion does not change the curvature of these two bands; thus, there is a band crossing between VBM and CBM in each *k* direction. Such band crossing phenomena can be predicted by *k*·*P* and group theory

Crossing in one of the *k* directions or in both *k*_*x*_ and *k*_*y*_ directions is critical to an indirect band gap of the system which will be further discussed at the end of the later subsection.

### SOC Gap and Indirect Band Gap of a Topological Insulator

In this subsection, at first, we show how SOC can open a band gap at crossing point. Then, we give the evidence proving the existence of TI phase in antimonene and show how the SOC gap depends on strain. Finally, we discuss how to avoid an indirect band gap that accompanies with the band inversion of a TI.

The last subsection has already shown that strain can induce band inversion at *Γ* point and causes a band crossing point in *k*_*x*_ or *k*_*y*_ direct.

Treating SOC as a perturbative term, and considering a two-band modeling Hamiltonian at the band crossing point:

7 $$  H= \left(\begin{array}{cc} E_{k\cdot P} & A \\ A^{*} & E_{k\cdot P}^{\prime\prime} \\ \end{array}\right),  $$

where *E*_*k*·*P*_ and $ E_{k\cdot P}^{\prime \prime } $ are the bands’ energy without considering SOC, and *A* is the SOC term. At the crossing point, these two bands are degenerated; thus, $ E_{k\cdot P} = E_{k\cdot P}^{\prime \prime } $. The energy eigenvalues of Eq. 7 are *E*_*k*·*P*_±|*A*|, which means these two bands open a gap at the crossing point, and the magnitude of the gap is 2|*A*| being proportional to the strength of SOC.

Since the band gap is opened by SOC, strained antimonene can be insulating in bulk after the band inversion (as shown in Fig. 3). As strained antimonene has central inversion symmetry and the band inversion at *Γ* point exchanges the opposite parity of VBM and CBM, thus, strained antimonene may have topological insulator phase.

**Fig. 3:** Band structures before (*left*) and after (*right*) the band inversion. *Positive strain* indicates expansion and *negative strain* indicates compression. All energies are referenced to Fermi level. The *dashed lines* are merely a guide for viewing the energy shifts of each band. The *signs* (+, −) (associate with band 1, 3) indicate the parities of the wavefunctions of *Γ* point states. The band structures show that, when considering SOC, antimonene can remain in insulator phase after the band inversion

It is well known that the nature of topology phase of a system can be examined by its parity product of all the time reversal invariant (TRI) momentum points. Therefore, we calculate the *Z*_2_ index of the system to confirm the topological insulator phase [14].

The *Z*_2_ index *ν* can be calculated by the following equation,

8 $$  (-1)^{\nu} = \prod\limits_{i} \Theta_{i},  $$

where

9 $$  \Theta_{i} = \prod\limits_{n=1}^{N} \vartheta_{2n} (\Gamma_{i}),  $$

in which 2N is total number of occupied bands, and *𝜗*_2*n*_(*Γ*_*i*_) is the parity eigenvalue of the 2n-th occupied band at the time reversal invariant momentum *Γ*_*i*_. Our first-principles calculations show that the *Z*_2_ index is zero before the band inversion. Just after the band inversion, *Z*_2_ invariant changes from 0 to 1, meaning that the system is changed to be a TI.

Without considering SOC, strained antimonene has a band crossing between VBM and CBM at some *k*=*k*_*c*_ point after the band inversion and such a crossing point can be located at a larger *k* point while the *Γ* point inversed band gap (GPIBG) is larger (as shown in Fig. 4). Furthermore, since the SOC term has *k*-dependent part (as shown in Eq. 4), the strength of SOC |*A*| is *k*-dependent. While considering SOC which opens a band gap at the crossing point, the magnitude of the SOC gap depends on the strength of SOC which increases as the magnitude of *k*_*c*_ increases. Since the *Γ* point inversed band gap (GPIBG) can be tuned by strain, the SOC gap at *k*_*c*_ can simultaneously be enhanced by strain.

**Fig. 4:** *k*_*c*_ is the crossing point of VBM and CBM. The band structures in **a** and **b** show that a larger strain can induce a larger *Γ* point inversed band gap (GPIBG). The magnitude of *k*_*c*_ will be increased as GPIBG becomes larger. Since the strength of SOC |*A*| increases as *k* does, thus, the magnitude of SOC gap increases as *k*_*c*_ does. Therefore, the SOC gap can be enhanced by strain. **c** The band structures of strained antimonene with the other high symmetry points. Due to the anisotropic property of *α*-phase antimonene, the *x* direction crossing point locates at a higher energy level than that of in *y* direction and causes an indirect bulk band gap. While the strain increases, the SOC gap is increased, but the energy difference between *x* direction crossing point and *y* direction crossing point is increased too. Consequently, the bulk band gap will close again when the strain becomes too large. **d** The magnitude of the SOC gap in *k*_*y*_ direction and the indirect bulk band gap of antimonene against different values of *y* direction strain (*x* direction strain is +14 *%*); negative indirect bulk band gaps indicate that the indirect bulk band gap of antimonene is closed and the system turns into a metal

Unfortunately, the magnitude of SOC gap is not the value of bulk band gap of antimonene. Due to the anisotropic property of *α*-phase antimonene, the *x* direction crossing point locates at a higher energy level than that in *y* direction and causes an indirect bulk band gap. When the strain increases, the SOC gap is increased, but the energy difference between *x* direction crossing point and *y* direction crossing point is increased too. Consequently, the bulk band gap will eventually close again when the strain becomes too large (as shown in Fig. 4 c, d).

There are two ways to avoid such an indirect band gap closing. One is applying strain on a system of more isotropic. The other is applying strain on an anisotropic system whose VBM and CBM are coupled to each other in one of the *k* directions by non-SOC *k*·*P* term. One of the examples is applying in-plane isotropic strain on antimonene. In-plane isotropic strain can cause a band inversion between band 2 and band 3. As shown in Eq. 5, band 2 and band 3 are coupled in *k*_*x*_ direction while decoupled in *k*_*y*_ direction. Thus, there are only one crossing point between band 2 and band 3 after the band inversion. Therefore, the band inversion does not cause an indirect band gap around the *Γ* point (as shown in Fig. 5). Even though the in-plane isotropic strain turns antimonene to be a metal before causing the band inversion between band 2 and band 3 (as shown in Fig. 2 a) and consequently TI phase is forbidden in this case, there are other cases that, in other materials or with other band inversion mechanisms, transition to metal phase can be avoided. An example in reference [44] shows that electric field can induce a band inversion between VBM and CBM as the VBM and CBM are coupled to each other in one of the *k* directions by non-SOC *k*·*P* term, an indirect band gap accompanying with the band inversion is avoided even though the system has an anisotropic property. This example implies that transition to metal phase can be avoided in some cases.

**Fig. 5:** The band structure of strained antimonene. **a** Without SOC. **b** With SOC. The in-plane isotropic strain causes a band inversion between band 2 and band 3. Since band 2 and band 3 are decoupled in *k*_*y*_ direction but coupled in *k*_*x*_ direction by non-SOC *k*·*P* term, band inversion between CBM and VBM cause only one crossing point. After considering SOC, a band gap open at the crossing point. Because there are only one crossing point, this band inversion does not accompany with an indirect band gap around the *Γ* point which is different with the band inversion between band 1 and band 3 (as shown in Fig. 4 c)

Based on this band analysis of antimonene, we suggest the mechanism of inducing strain-enhanced SOC gap should apply to systems of more isotropic or to other anisotropic systems whose VBM and CBM are coupled to each other in one of the *k* directions by non-SOC *k*·*P* term for achieving the goal of searching large bulk band gap TI.

There are some reports that some large bulk band gap TI systems are stable under strain and can be candidate materials for spintronics device [1, 3, 8]. Even though antimonene is not stable under large strain, the methodology of finding lager band gap spintronics device is still valid; a further study of finding those large band gap TI can be accelerated with the help of our proposed band analysis.

## Conclusions

In this paper, we analyze antimonene with *k*·*P* theory and find that without considering SOC, strain-induced *Γ* point band inversion would cause band crossing between VBM and CBM and the system simply turns into metallic state. With SOC included, band gap opens at the crossing point in a way that antimonene remains insulating after the band inversion. Then, we use *Z*_2_ invariant to prove that while strained antimonene remains in insulator phase after the band inversion, antimonene has a topological non-trivial phase.

Furthermore, because strain can enhance the spin-orbit coupling between VBM and CBM at the crossing point, the SOC gap increases as the strain does. With such a mechanism, the magnitude of the SOC gap no longer depends on the atomic order only. Thus, searching large bulk band gap TI among light atoms becomes possible, though the SOC gap is not always the bulk band gap of a TI.

The *k*·*P* theory indicates that, in an anisotropic system, the band inversion of a TI phase transition will accompany with an indirect band gap if VBM and CBM cannot couple to each other by non-SOC *k*·*P* term. The magnitude of such an indirect band gap decreases as the strain increases. With the indirect band gap, the SOC gap cannot be the bulk band gap. Therefore, the indirect band gap should be avoided. Inducing strain-enhanced SOC gap should be promoted to more isotropic systems or to other anisotropic systems whose VBM and CBM are coupled to each other in one of the *k* directions by non-SOC *k*·*P* term.
